# Increased constitutive αSMA and Smad2/3 expression in idiopathic pulmonary fibrosis myofibroblasts is K_Ca_3.1-dependent

**DOI:** 10.1186/s12931-014-0155-5

**Published:** 2014-12-05

**Authors:** Katy M Roach, Heike Wulff, Carol Feghali-Bostwick, Yassine Amrani, Peter Bradding

**Affiliations:** Department of Infection, Immunity and Inflammation, Institute for Lung Health, University of Leicester, Leicester, LE3 9QP UK; Department of Pharmacology, University of California, Davis, California 95616 USA; Department of Medicine, Division of Rheumatology and Immunology, University of South Carolina, Columbia, USA

**Keywords:** Idiopathic pulmonary fibrosis (IPF), Fibrosis, Lung, Myofibroblast, K_Ca_3.1, Ion channel, Differentiation, Smad 2, Smad 3

## Abstract

**Background:**

Idiopathic pulmonary fibrosis is a common and invariably fatal disease with limited therapeutic options. Ca^2+^-activated K_Ca_3.1 potassium channels play a key role in promoting TGFβ1 and bFGF-dependent profibrotic responses in human lung myofibroblasts (HLMFs). We hypothesised that K_Ca_3.1 channel-dependent cell processes regulate HLMF αSMA expression via Smad2/3 signalling pathways.

**Methods:**

In this study we have compared the phenotype of HLMFs derived from non-fibrotic healthy control lungs (NFC) with cells derived from IPF lungs. HLMFs grown *in vitro* were examined for αSMA expression by immunofluorescence (IF), RT-PCR and flow cytommetry. Basal Smad2/3 signalling was examined by RT-PCR, western blot and immunofluorescence. Two specific and distinct K_Ca_3.1 blockers (TRAM-34 200 nM and ICA-17043 [Senicapoc] 100 nM) were used to determine their effects on HLMF differentiation and the Smad2/3 signalling pathways.

**Results:**

IPF-derived HLMFs demonstrated increased constitutive expression of both α-smooth muscle actin (αSMA) and actin stress fibres, indicative of greater myofibroblast differentiation. This was associated with increased constitutive Smad2/3 mRNA and protein expression, and increased Smad2/3 nuclear localisation. The increased Smad2/3 nuclear localisation was inhibited by removing extracellular Ca^2+^ or blocking K_Ca_3.1 ion channels with selective K_Ca_3.1 blockers (TRAM-34, ICA-17043). This was accompanied by de-differentiation of IPF-derived HLMFs towards a quiescent fibroblast phenotype as demonstrated by reduced αSMA expression and reduced actin stress fibre formation.

**Conclusions:**

Taken together, these data suggest that Ca^2+^- and K_Ca_3.1-dependent processes facilitate “constitutive” Smad2/3 signalling in IPF-derived fibroblasts, and thus promote fibroblast to myofibroblast differentiation. Importantly, inhibiting K_Ca_3.1 channels reverses this process. Targeting K_Ca_3.1 may therefore provide a novel and effective approach for the treatment of IPF and there is the potential for the rapid translation of K_Ca_3.1-directed therapy to the clinic.

## Introduction

Idiopathic pulmonary fibrosis (IPF) has an unknown etiology [1] and is marked by progressive lung fibrosis leading to respiratory failure. The pathogenic mechanisms involved in its initiation and progression are poorly understood [2] and there are limited therapeutic options with poor efficacy [3,4]. Prognosis is bleak with a median survival of only 3 years, worse than many cancers [5]. IPF patients present with a mean age of between 60 to 65 years at diagnosis [4]. In the USA the overall incidence of IPF is 16 per 100,000 person-years [2] and the incidence is increasing by 11% annually in the UK [6]. The most favoured hypothesis regarding its development is that on-going multiple, microscopic, isolated episodes of alveoli epithelial injury lead to an abnormal wound healing response involving fibrotic repair mechanisms [7].

Fibroblasts are mesenchymal cells that serve a critical role in both normal and fibrotic repair processes, which when activated, become differentiated, highly secretory and contractile smooth muscle-like cells termed myofibroblasts [8]. Expression of alpha smooth muscle actin (αSMA) and αSMA-containing stress fibres is the hallmark of these cells [9-12]. IPF evolves from dysfunctional interactions between the injured epithelium and fibroblasts which lead to pathologic lesions called fibroblast foci, which are comprised of activated myofibroblasts [13]. In their activated state, myofibroblasts are the primary cell responsible for the synthesis, secretion and remodelling of the extracellular matrix in IPF [14]. The human lung myofibroblast (HLMF) is therefore an attractive target for the treatment of IPF.

αSMA is a key protein expressed by HLMFs as compared to quiescent fibroblasts [15], and contributes to the formation of characteristic HLMF contractile stress fibres [8,16,17]. αSMA expression and stress fibre formation in myofibroblasts is regulated in part by the TGFβ1/Smad signalling pathway [18,19]. Smads are intracellular proteins which transduce TGFβ1-dependent signals. Following binding of TGFβ1 to the TGFβRII, Smad2/3 are phosphorylated and form hetero-oligomeric complexes with Smad 4, leading to nuclear translocation and the regulation of gene transcription [20]. They therefore regulate many biological effects in HLMFs that are under the control of TGFβ1, including collagen secretion, proliferation, differentiation and contraction [18-21].

Ion channels are attractive therapeutic targets for many chronic diseases including fibrosis. Activated intermediate conductance Ca^2+^-activated K^+^ channels promote several pro-fibrotic processes in HLMFs such as basic fibroblast growth factor (bFGF)-dependent proliferation, and TGFβ1-dependent wound healing, collagen secretion and contraction [22]. K_Ca_3.1 activity was also shown to contribute to the upregulation of αSMA in response to TGFβ1 through the enhancement of Smad phosphorylation [23], and contributed to diabetic [24] and surgically-induced kidney fibrosis in rodents [25]. However, much of the research published to-date has focussed on the activity of myofibroblasts following TGFβ1 stimulation, and there are few studies investigating basal signalling differences between non fibrotic control (NFC) and IPF-derived myofibroblasts. Previously, IPF-derived HLMFs demonstrated significantly higher constitutive αSMA [26] and functional K_Ca_3.1 channel expression [22] compared to NFC-derived cells. However, whether these basal increases in αSMA in IPF-derived HLMFs are due to altered constitutive Smad pathway signalling or K_Ca_3.1 activity is not known.

We therefore hypothesized that Smad2/3 signalling is increased at baseline in IPF-derived HLMFs compared to NFC cells, and if true, that this would be susceptible to K_Ca_3.1 channel inhibition. We therefore investigated constitutive Smad2/3 nuclear localisation and αSMA expression in NFC- and IPF-derived HLMFs, and the role of K_Ca_3.1 ion channels in these processes.

## Materials and methods

### Human lung myofibroblast isolation and culture

Non-fibrotic control (NFC) HLMFs were derived from healthy areas of lung from patients undergoing lung resection for carcinoma at Glenfield Hospital, Leicester, UK. No morphological evidence of disease was found in the tissue samples used for HLMF isolation. IPF HLMFs were derived from patients undergoing lung biopsy for diagnostic purposes at the University of Pittsburgh Medical Center, USA, and were shown to have UIP on histological examination. Myofibroblasts were grown from explanted lung tissue from both sources under identical conditions, using DMEM supplemented with 10% FBS, antibiotic/antimycotic agents and non-essential amino acids [27,28]. The cells were cultured at 37°C in 5% CO_2_/95% air. Cells were studied at passages 4–5 for functional studies. HLMFs were characterised as previously described [22]. All NFC patients gave informed written consent and the study was approved by the National Research Ethics Service (references 07/MRE08/42 and 10/H0402/12). Written informed consent was also obtained from all IPF subjects, in accordance with the responsible University of Pittsburgh Institutional Review Board.

### Human myofibroblast characterisation

Human myofibroblasts were harvested from 80-90% confluent monolayers with 0.1% trypsin/0.1% EDTA. Cells were seeded into 8-well chamber slides, grown to confluence, and to confirm a myofibroblast population the cells were immunostained using the following antibodies: FITC-conjugated mouse monoclonal anti-α-smooth muscle actin (αSMA) (F3777, 10 μg/ml, Sigma-Aldrich, Poole, Dorset, UK); mouse monoclonal anti-fibroblast surface protein(FSP)(F4771, 4 μg/ml, Sigma-Aldrich); mouse monoclonal anti-fibroblast antigen THY-1 (CP28, 3 μg/ml, Calbiochem, San Diego, CA; rabbit polyclonal collagen type 1 (550346, 20 μg/ml, Millipore, Watford, UK), isotype control rabbit IgG (20 μg/ml). To detect the presence of contaminating cells the following antibodies were used; monoclonal mouse CD68 antibody (6.4 μg/ml, Dako) to detect the presence of macrophages, mast cells and monocytes; mouse monoclonal CD3 (4.5 mg/ml Dako) to detect T-cells, and mouse monoclonal CD34 R-PE antibody (0.5 μg/ml, Catlag) was also used to detect progenitor cells. Secondary antibodies labelled with FITC or R-PE (F0313, Dako) were applied and the cells counterstained with 4′,6-diamidino-2-phenylindole (DAPI, Sigma-Aldrich). All isotype controls were negative. Cells were mounted with fluorescent mounting medium and cover-slipped. The results confirmed that the cells isolated were of myofibroblast-rich population of cells (99%), with no contaminating cells identified. Full details, results and accompanying images have been previously published in Roach et al. [22].

### Immunofluorescence

HLMFs were grown on 8-well chamber slides and serum-starved for 24 hours prior to the experiment. The cells were then treated for 24 hours with either 0.1% DMSO, TRAM-34 (20 and 200 nM) or ICA-17043 (10 and 100 nM). Cells were then immunostained as described previously [22] using FITC-conjugated mouse monoclonal anti-α-SMA (F3777, 10 μg/ml, Sigma-Aldrich, Poole, Dorset, UK) and isotype control FITC-conjugated mouse IgG_2a_ (X0933, 10 μg/ml, Dako, Ely, UK). K_Ca_3.1 expression was examined by immunofluorescence using rabbit polyclonal anti-K_Ca_3.1 (AV35098, 5 μg/ml, Sigma) and appropriate isotype control. Secondary antibodies labelled with FITC (F0313, Dako) were applied and the cells counterstained with 4′,6-diamidino-2-phenylindole (DAPI, Sigma-Aldrich). Cells were mounted with fluorescent mounting medium and cover-slipped. Original images were captured on an epifluorescent microscope (Olympus BX50, Olympus UK Ltd, Southend–on-sea); grey scale intensity was examined using Cell F imaging software (Olympus UK Ltd). Matched exposures were used for isotype controls.

Actin stress fibres were calculated using a specialised macro on image J designed by Dr Kees Straatman, University of Leicester. The macro is capable of providing a quantitative, unbiased score of the number of stress fibres per individual cell by determining the fluctuations of grey scale intensity created by the αSMA staining within the stress fibres.

### Flow cytometry

Cells were grown on T25 flasks and serum-starved for 24 hours prior to the experiment. The myofibroblasts were incubated for 24 hours in the presence of 0.1% DMSO control, TRAM-34 (200 nM) or ICA-17043 (100 nM). Cells were detached using 0.1% trypsin/0.1% EDTA, washed then fixed and permeabilised in 4% paraformaldehyde plus 0.1% saponin (Sigma) respectively for 20 minutes on ice. Myofibroblasts were labelled with FITC-conjugated mouse monoclonal anti-α-smooth muscle actin (sigma) or isotype control FITC-conjugated mouse IgG_2a_. Secondary antibodies labelled with FITC (F0313, Dako) were applied. Analysis was performed using single colour flow cytometry on a FACScan (BD, UK).

### Smad nuclear localisation

HLMFs were grown on 8-well chamber slides and serum-starved for 24 hours prior to the experiment. The cells were then stimulated with TGFβ1 (10 ng/ml) in the presence of either 0.1% DMSO control, TRAM-34 (200 nM), ICA-17043 (100 nM) or Ca^2+^ free media. After 1 hour cells were immunostained using rabbit monoclonal anti-Smad2/3 (0.174 μg/ml, Cell Signalling). Secondary antibody labelled with FITC (F0313, Dako) was applied and the cells counterstained with DAPI (Sigma-Aldrich). Cells were mounted with fluorescent mounting medium and cover-slipped. Images were analysed as above. The intensity of nuclear Smad2/3 staining was quantified by measuring the grey scale intensity of DAPI positive nuclei to whole cell staining.

### Western blot for Smad proteins

Cells were grown in T75 flasks, serum starved for 24 hours, and then incubated with either 0.1% DMSO control, TRAM-34 (200 nM), ICA-17043 (100 nM) or Ca^2+^ free media for 1 hour. Cells were detached with 0.1% Trypsin/EDTA and washed. Protein was isolated using the RIPA buffer lysis system (Santa Cruz, Germany) and total protein concentration was determined using the DC Bio-Rad protein Assay (Bio-Rad, UK). 30 μg of protein was resolved using 10% Mini-Protean TGX precast gels (Bio-Rad) and then transferred to an immunobilon-P polyvinylidene difluoride membrane, using Trans-blot Turbo transfer packs (Bio-Rad). Membranes were blocked with 5% milk and incubated with rabbit monoclonal anti-phospho-Smad2/3 (0.231 μg/ml, Cell Signalling, USA), rabbit polyclonal anti-Smad2/3 (0.0087 μg/ml, Cell Signalling), mouse monoclonal anti-TATA binding protein (TBP) (1 μg/ml, Abcam), or mouse monoclonal anti-β-actin antibody (0.2 μg/ml, SantaCruz). Protein bands were identified by horseradish peroxidase-conjugated secondary antibody and enhanced chemiluminescence reagent (Amersham, UK). Immunolabelled proteins were visualized using ImageQuant LAS 4000 (GE Healthcare Life Sciences, UK).

### Nuclear fraction

NFC and IPF-derived HLMFs were grown in T75 flasks, serum starved for 24 hours, then detached with 0.1% Trypsin/EDTA and washed. Nuclear and cytoplasmic extracts were isolated using the Nuclear Extract Kit (Abcam, ab113474). Protein concentrations of both nuclear and cytoplasmic extract was then was isolated using the RIPA buffer lysis system determined using the DC Bio-Rad protein Assay. Western blot was then performed as described above.

### qRT-PCR

Myofibroblast RNA was isolated using the RNeasy Plus Kit (Qiagen, West Sussex, UK) according to the manufacturer’s instructions. Primers were designed for Smad2 , forward CGTCCATCTTGCCATTCACG and reverse CTCAAGCTCATCTAATCGTCCTG, product size 182 bp from NCB1 Reference sequence NM_005901.5; and Smad3, forward GCGTGCGGCTCTACTACATC and reverse GCACATTCGGGTCAACTGGTA product size 233 bp from reference sequence NM_005902.3 β-actin primers were analysed using gene-specific Quantitect Primer Assay primers (Qiagen, Germany), HS_ACTB_1_SG. All expression data were normalized to β-actin and corrected using the reference dye ROX. Gene expression was quantified by real-time PCR using the Brilliant SYBR Green QRT-PCR 1-Step Master Mix (Strategene, The Netherlands). PCR products were run on a 1.5% agarose gel to confirm the product amplified was the correct size, and each of the products were sequenced to confirm the specificity of the primers.

### Statistical analysis

Experiments from an individual donor were performed either in duplicate or triplicate and a mean value was derived for each condition. Cells from 8 IPF and 8 NFC donors were used, and the number of donors used for each experimental condition is stated in the text and/or figure legends. Data distribution across donors was tested for normality using the Kolmogorov-Smirnov test. For parametric data the 1-way ANOVA or repeated measures ANOVA for across-group comparisons was used followed by the appropriate multiple comparison post hoc test; otherwise an unpaired or paired t-test was used. For non-parametric data the Friedman test was used for across group comparisons followed by the appropriate multiple comparison post hoc test, or the Mann Whitney U test was used where there were two unpaired groups. GraphPad Prism for windows (version 6, GraphPad Software, San Diego California USA) was used for these analyses. A value of P < 0.05 was taken to assume statistical significance and data are represented as mean (± SEM) or median (IQR).

## Results

### IPF myofibroblasts have increased basal αSMA expression and stress fibre formation

We and others have shown previously that fibroblasts grown from lung parenchyma express relatively high levels of αSMA and are contractile [22,29], in keeping with a myofibroblast phenotype. Here both NFC and IPF-derived HLMFs expressed αSMA protein, but this was significantly increased in IPF derived cells when assessed by immunofluorescent staining (P = 0.0111, Figure 1A and B), western blot analysis (P = 0.0026, Figure 1C and D) and flow cytometry, P = 0.0159 (Figures 1E and F).

**Figure 1:** **IPF myofibroblasts have increased basal αSMA expression and stress fibre formation. (A)** HLMF αSMA expression was measured by grey scale intensity in n = 7 NFC and n = 7 IPF donors; a minimum of 10 random cells were measured in one field for each donor. IPF HLMF’s had significantly higher intensity of αSMA in comparison to NFC donors P = 0.0111, Mann–Whitney. **(B)** Immunofluorescent images displaying αSMA staining and actin stress fibers in the cytoplasmic matrix. **(C and D)** Western blot analysis of αSMA expression in NFC (n = 3) and IPF-derived (n = 3) HLMFs, **P = 0.0026. The detected band was at the correct molecular weight of 42 kDa for αSMA **(E and F)** the mean fluorescent intensity (MFI) of αSMA expression assessed by flow cytometry. IPF (n = 4) donors showed significantly higher expression than NFC (n = 4), P = 0.0159. **(G)** Illustration of how the αSMA stress fibres were assessed. A macro recorded the number of fibres per individual cell. Each fibre represents a peak in grey value and the number of peaks equating to the number of stress fibres was then counted per cell. A minimum of 10 cells were measured per donor. **(H)** The results show that the number of actin stress fibres were significantly higher in IPF (n = 8) donors in comparison to NFC (n = 8) donors P = 0.0437 (Un-paired t-test). Results are presented as median ± IQR, #P < 0.05 (Mann–Whitney), or mean ± SEM *P < 0.05, **P < 0.01 (Unpaired t-test).

Both NFC and IPF-derived cells displayed cytosolic αSMA staining, but IPF-derived HLMFs displayed obvious αSMA-positive stress fibres. Immunofluorescent pictures were examined using an Image J macro which measured the numbers of stress fibres per cell, this is shown in Figure 1G. We found significantly more αSMA positive stress fibres in IPF-derived cells in comparison to NFC donors, P = 0.0437 (Figure 1H).

### IPF myofibroblasts have increased basal K_Ca_3.1 expression

Functional K_Ca_3.1 channels are increased in IPF-derived HLMFs [22]. We therefore examined the expression of K_Ca_3.1 by immunofluorescence and its relationship to αSMA expression. We found that IPF-derived HLMFs had a higher intensity of immunostaining than NFC cells, (Figure 2A and B), in keeping with previous patch clamp electrophysiology data [22]. Furthermore, K_Ca_3.1 expression correlated significantly with both basal αSMA expression, r = 0.79, P = 0.0176, and basal Smad2/3 localisation, r = 0.9245, P = 0.0029 in both NFC and IPF donors (Figure 2C and D).

**Figure 2:** **K**_**Ca**_ **3.1 protein expression in HLMFs. (A)** K_Ca_3.1 protein expression in HLMFs was measured using the grey scale intensity and was significantly higher in IPF (n = 4) in comparison to NFC-derived cells (n = 4), mean ± SEM, *P < 0.05 (Un-paired t-test). **(B)** Examples of K_Ca_3.1 immunofluorescent staining in both NFC and IPF donors. **(C)** The correlation between K_Ca_3.1 and αSMA expression in HLMFs, r = 0.798, P = 0.0176. **(D)** The correlation between K_Ca_3.1 and whole cell nuclear Smad expression in HLMFs, r = 0.925, p = 0.0029.

### Smad2/3 expression is greater in IPF-derived HLMFs

To elucidate the molecular mechanisms underlying the observed phenoytypic differences between NFC- and IPF-derived HLMFs we investigated the basal Smad2/3 content as Smad2/3 signalling is key for myofibroblast differentiation and αSMA gene transcription RT-PCR results confirmed that both Smad2 and Smad3 mRNA were significantly upregulated in IPF-derived HLMFs compared to NFC-derived cells, P = 0.0286 and P = 0.0286 respectively, Mann Whitney (Figure 3A and B). Smad3 mRNA was more highly expressed than Smad2 mRNA (Figure 3C).

**Figure 3:** **Total and nuclear Smad2 and Smad3 expression is significantly higher in IPF-derived HLMFs. (A)** Smad2 mRNA expression was examined by qRT-PCR in NFC (n = 4) and IPF (n = 4) myofibroblasts. IPF-derived HLMFs had significantly higher Smad2 mRNA at baseline in comparison to NFC-derived cells. **(B)** Similarly, Smad3 mRNA expression was significantly higher in IPF-derived HLMFs (n = 4) in comparison to NFC-derived cells (n = 4). **(C)** Smad3 mRNA expression was increased compared to Smad2 mRNA expression in both NFC and IPF-derived HLMFs.** (D and E)** Quantification of Western blot analysis showed that total Smad2/3 protein was increased in IPF-derived HLMFs in comparison to NFC-derived cells. Results were normalised to β-actin.** (F)** The proportion of total Smad2/3 nuclear staining to whole cell staining was measured in at least 10 cells in HLMFs from both NFC (n = 7) and IPF (n = 9) donors. IPF-derived HLMFs had a significantly higher proportion of Smad2/3 located in the nucleus compared to NFC-derived cells. **(G)** A representative illustration of total Smad2/3 expression assessed by immunofluorescence. **(H)** Representative Western blot analysis showing total Smad2/3 protein within the nucleus and cytoplasm of IPF and NFC-derived cells. TBP is localized to nuclear enriched fractions relative to cytoplasmic enriched fractions, similarly β-actin is localized to cytoplasmic enriched fractions relative to nuclear enriched fractions, N = nucleus, C = cytoplasm. Detected bands were at the correct molecular weight of 52 and 60 kDa for total Smad2 and Smad3 respectively, 38 kDa for TBP and 43 kDa for β-actin **(I)** Quantification of Western blot analysis confirmed that total Smad2/3 in the nuclear enriched fraction is significantly increased in IPF cells (n = 3) in comparison to NFC cells (n = 3). Results were normalized to TBP. **(J)** Similarly, total Smad2/3 in the cytoplasmic enriched fraction was increased in IPF cells (n = 3) in comparison to NFC-derived cells (n = 3). Results were normalized to β-actin. Results are represented as mean ± IQR #P < 0.05 (Mann Whitney) or mean ± SEM *P = 0.05 (Un-paired t-test).

Total Smad2/3 protein expression was significantly increased in IPF-derived HLMF donors compared to NFC-derived cells, P = 0.0294, unpaired t test (Figure 3D and E), although phosphorylated Smad2/3 was undetectable in both IPF and NFC-derived cells. Immunofluorescent staining revealed that constitutive Smad2/3 nuclear staining was significantly greater in IPF-derived HLMFs in comparison to NFC-derived cells, P = 0.0202, unpaired t test (Figure 3F and G). To confirm the observed increased nuclear staining of IPF-derived cells, Western blot was performed examining total Smad2/3 protein expression in the nuclear fraction and cytoplasmic extract of IPF and NFC-derived cells. Cytoplasmic and nuclear fractions were probed for the nuclear protein, TATA box binding protein (TBP) and β-actin to verify separation. As expected TBP was observed primarily in the nuclear protein enriched fractions, and served as a nuclear loading control for analysis. β-actin was observed primarily in the cytoplasmic protein enriched fractions and was used as the cytoplasmic loading control for subsequent analysis. The results demonstrate that IPF-derived HLMFs have significantly greater amounts of total Smad2/3 within the nucleus and cytoplasm in comparison to NFC HLMFs, P = 0.0488 and P = 0.0454 respectively (Figure 3H,I and J). This suggests that there may be increased constitutive Smad2/3 signalling in IPF-derived HLMFs.

### Constitutive Smad 2/3 expression is inhibited by K_Ca_3.1 blockers and is Ca^2+^ dependent

K_Ca_3.1 channel activity is important for profibrotic HLMF processes such as proliferation, contraction and collagen secretion [22]. Because the Smad2/3 pathway is a major regulator of αSMA and collagen secretion [18,19,30], we investigated whether the selective K_Ca_3.1 blockers TRAM-34 (20 and 200 nM)(Kd for TRAM-34 is 20 nM) [31] and ICA-17043 (10 and 100 nM)(Kd for ICA-17043 is 10 nM) [32] have inhibitory effects on the basal nuclear translocation of Smad2/3 in HLMFs. Using immunofluorescence we found a significant reduction in the amount of Smad2/3 in the nucleus of HLMFs following 1 hour incubation with TRAM-34 200 nM, P = 0.0008 (Figure 4A and B). Similarly, ICA-17043 100 nM significantly inhibited Smad2/3 nuclear staining, P = 0.0003 (Figure 4C and D).

**Figure 4:** **Basal nuclear total Smad2/3 expression is significantly attenuated by K**_**Ca**_ **3.1 blockers. (A)** Constitutive nuclear Smad2/3 expression was significantly attenuated by the K_Ca_3.1 blocker TRAM-34 (200 nM) (NFC n = 5 [triangles] and IPF n = 6 [circles] (data pooled for statistical analysis, at least 10 cells were measured per donor). **(B)** Immunofluorescent images depict the reduced nuclear staining following 1 hour of incubation with TRAM-34. **(C and D)** Similarly, ICA-17043 (100 nM) significantly reduced the proportion of total Smad2/3 staining within the nuclei of HLMFs after a 1 hour incubation. Results are represented as mean ± SEM, *P < 0.05 (Paired t-test).

K_Ca_3.1 channel blockade depolarises the plasma membrane and thereby reduces receptor-dependent rises in intracellular Ca^2+^ concentrations in many cell types including HLMFs [22,33-36]. If Ca^2+^ signalling is mechanistically important for the effects of K_Ca_3.1 blockers on constitutive Smad2/3 nuclear translocation, lowering the extracellular Ca^2+^ concentration should also inhibit nuclear translocation. Incubating HLMFs for 1 hour in Ca^2+^-free media significantly reduced the amount of Smad2/3 in the nuclei compared to cells incubated in media containing normal external Ca^2+^ (1.8 mM), P = 0.0114 (Figure 5A and B). This suggests that the enhancement of Ca^2+^-influx by K_Ca_3.1 channels is an essential requirement for the efficient nuclear translocation of Smad2/3 and subsequent transcription and expression of αSMA.

**Figure 5:** **Smad2/3 nuclear translocation is Ca** ^**2+**^ **dependent. (A)** When HLMFs were incubated with Ca^2+^-free medium for 1 hour there was a significant reduction in the amount of Smad2/3 located in the nucleus, NFC n = 3 and IPF n = 3 (a minimum of 10 random cells were measured in one field for each donor, data pooled for NFC and IPF). **(B)** Representative immunofluorescent staining demonstrating the attenuated nuclear expression of Smad2/3 in Ca^2+^-free medium. Results are represented as mean ± SEM, *P < 0.05 (Paired t-test).

### αSMA expression in HLMF is inhibited by K_Ca_3.1 blockers

Next we assessed whether the inhibition of constitutive Smad2/3 nuclear translocation following K_Ca_3.1 block was associated with a reduction in αSMA expression and thus de-differentiation of HLMFs back towards a fibroblast phenotype. We therefore incubated both NFC- and IPF-derived HLMFs with the TRAM-34 (20 and 200 nM) and ICA-17043 (10 and 100 nM) [32] for 24 hours. No significant differences between NFC and IPF donors were seen in response to K_Ca_3.1 blockers so statistics were performed on pooled data. Both TRAM-34 and ICA-17043 dose-dependently inhibited the constitutive expression of HLMF αSMA assessed by immunofluorescent staining, P < 0.0001 (2-way ANOVA) (Figure 6A-C). No inhibition of αSMA expression was seen with two structurally related molecules without channel blocking activity, TRAM-85 and TRAM-7 [31] (Figure 6D). Decreases in constitutive αSMA expression were also confirmed by flow cytometry(P = 0.0078 for TRAM-34 and P = 0.0391 for ICA-17043) (Figure 6E and F).

**Figure 6:** **K**_**Ca**_ **3.1 channel inhibition reduces constitutive HLMF αSMA expression. (A)** The percentage of cells expressing αSMA was dose-dependently decreased by TRAM-34 in NFC (n = 3) and IPF (n = 3)-derived HLMFs (a minimum of 10 random cells were measured in one field for each donor, data for NFC and IPF pooled for statistical analysis). **(B)** Similarly, αSMA expression was dose-dependently attenuated by ICA-17043 in NFC (n = 5) and IPF (n = 3)-derived HLMFs (data pooled for statistical analysis). No differences were evident between NFC and IPF-derived cells. **(C)** Representative immunofluorescent images illustrating decreased αSMA expression in the actin filaments and cytoplasm following K_Ca_3.1 inhibition with TRAM-34 (20 nM and 200 nM) and ICA-17043 (10 nM and 100 nM). **(D)** Two structurally related molecules without channel blocking activity, TRAM-85 and TRAM-7, did not reduce constitutive αSMA expression in NFC (n = 2) and IPF (n = 2)-derived HLMFs (data pooled, P < 0.999 and p = 0.1244 respectively). **(E and F)** The mean fluorescent intensity (MFI) of constitutive αSMA expression was also assessed by flow cytometry. TRAM-34 (200 nM) **(E)**, and ICA-17043 (100 nM) **(F)**, again reduced αSMA expression significantly in NFC (n = 4) and IPF (n = 4)-derived HLMFs (data pooled for statistical analysis). Results are represented as mean ± SEM ***P < 0.0001 (2 way ANOVA corrected by Dunnetts multiple comparison test) or median ± IQR #P < 0.05 and ##P < 0.01 (Wilcoxon signed rank test).

### αSMA stress fibres in HLMF are reduced by K_Ca_3.1 blockers

Following K_Ca_3.1 inhibition the number of actin stress fibres in both NFC and IPF-derived HLMFs were dose-dependently inhibited by TRAM-34 (20 nM and 200 nM), P = 0.0235 and ICA-17043 (10 nM and 100 nM), P = 0.0095, (Figure 7A and B). Thus not only is cytosolic αSMA staining inhibited by K_Ca_3.1 channel blockers but also αSMA stress fibres, suggesting a phenotypic transition from a myofibroblast into a more fibroblast-like phenotype.

**Figure 7:** **HLMF αSMA stress fibres are significantly attenuated by K**_**Ca**_ **3.1 blockers. (A)** TRAM-34 dose-dependently decreased the number of actin stress fibres (NFC n = 3 and IPF n = 3, data pooled for statistical analysis). **(B)** ICA-17043 dose-dependently decreased the number of actin stress fibres (NFC n = 5 and IPF n = 3, data pooled for statistical analysis). No difference in response to the K_Ca_3.1 blockers were seen between NFC and IPF donors. Results are represented as mean ± SEM *P < 0.05, **P < 0.01 (2 Way ANOVA corrected by Sidaks multiple comparisons test).

## Discussion

We have demonstrated that IPF-derived HLMFs constitutively overexpress αSMA and actin stress fibres together with an increase in constitutive Smad2/3 nuclear localisation when compared to NFC cells. The increased constitutive Smad2/3 nuclear localisation was heavily reliant on the presence of extracellular Ca^2+^, and was inhibited by selective K_Ca_3.1 ion channel blockers. Taken together, these data suggest that increased basal Ca^2+^- and K_Ca_3.1-dependent processes facilitate “constitutive” Smad2/3 signalling in IPF-derived fibroblasts, and thus promote fibroblast to myofibroblast differentiation. Importantly, inhibiting K_Ca_3.1 channels reversed this process.

Phenotypically both NFC and IPF-derived human lung parenchymal fibroblasts in culture demonstrate the classic fibroblast-like elongated morphology [21,22,37]. Previous work has shown that healthy lung parenchymal fibroblasts express high levels of αSMA and display upregulated genes associated with actin binding and cytoskeletal organisation together with up-regulation of activated Smad2 and Smad3 when compared to airway fibroblasts from the same donors [21]. These cultured lung parenchymal fibroblasts therefore have features of a myofibroblast phenotype, hence we describe them as HLMFs. Of note, IPF-derived HLMFs express higher concentrations of αSMA than cells from healthy lung [26,38], a finding we have confirmed here. In addition to this, we found that IPF-derived cells exhibited increased actin stress fibre formation and cytoskeletal organisation compared to NFC cells. We also found that IPF-derived HLMFs, without TGFβ1 stimulation, have significantly higher constitutive total Smad2/3 protein expression, greater Smad2/3 expression within the nucleus and higher Smad2 and Smad3 mRNA expression when compared to NFC control cells. Smad3 in particular was implicated in driving the myofibroblast phenotype in healthy parenchymal HLMFs [21], and while we found that both Smad2 and Smad3 mRNA were increased in IPF-derived HLMFs, Smad3 mRNA was significantly higher than Smad2 in both NFC and IPF-derived cells. This supports the work of Zhou et al. [21], but shows that differential Smad2 versus Smad3 mRNA expression persists in IPF-derived cells. Thus while healthy parenchymal lung fibroblasts exhibit features of a myofibroblast phenotype, this is significantly more pronounced in IPF-derived myofibroblasts.

The mechanism behind this increased constitutive myofibroblast differentiation in IPF-derived cells is unclear and potentially multi-factorial. That such a phenotypic difference persists for several passages in cell culture suggests that genetic or epigenetic factors may contribute [39]. Whether pre-programmed by genetics, or re-programmed by epigenetics, IPF-derived HLMFs clearly have the potential to perpetuate the fibrotic process. Reversing this pro-fibrotic phenotype is therefore an important goal therapeutically.

Irrespective of the point from where pathological HLMF differentiation occurs in IPF, we have shown that K_Ca_3.1 channels play a key role in this process. By patch clamp electrophysiology we have shown previously that functional K_Ca_3.1 ion channels are increased in IPF-derived HLMFs [22], and we found increased K_Ca_3.1 ion channel protein in this study. Importantly, we have shown here that blocking K_Ca_3.1 channels has the unique ability to de-differentiate HLMFs towards a fibroblast phenotype as indicated by a marked reduction in αSMA protein and stress fibre formation. This appears to operate via Ca^2+^-dependent processes as the reduction in constitutive nuclear Smad2/3 expression induced by K_Ca_3.1 blockers was mimicked by removing extracellular Ca^2+^, and K_Ca_3.1 channel activity is known to influence intracellular Ca^2+^ concentrations in many cell types [34,35,40-42]. For example, we demonstrated previously that K_Ca_3.1 activity is required for a rise in intracellular Ca^2+^ that occurs following exposure of HLMFs to TGFβ1 [22].

Previous studies have focused mainly on TGFβ1-dependent Smad2/3 processes and have been contradictory with regards to the role of Ca^2+^. A study on oesteoblasts showed that a TGFβ1-dependent Ca^2+^ signal was not required for Smad2 phosphorylation [43] where as in kidney fibroblasts, TGFβ1-dependent Smad function was controlled directly by Ca^2+^-calmodulin [44]. We found that constitutive Smad2/3 nuclear localisation is highly dependent on Ca^2+^ and K_Ca_3.1 channel activity. This suggests that the contribution of Ca^2+^ signals and K_Ca_3.1 activity to Smad2/3 signalling may be cell-specific. This well documented heterogeneity in fibroblast biology highlights the importance of studying cells from the relevant species and tissue of interest. Thus these data from primary IPF-derived HLMFs demonstrate the potential of K_Ca_3.1 as a target for IPF.

The increased nuclear localisation of Smad2/3 in IPF-derived HLMFs in association with increased αSMA actin and K_Ca_3.1 expression, and the parallel reductions in Smad2/3 nuclear localisation and αSMA expression following K_Ca_3.1 blockade, suggest that Smad2/3 signalling is likely to be increased constitutively in IPF-derived cells. However, we were unable to observe phosphoSmad2/3 in the cytoplasm or nucleus. Under these basal conditions, phosphoSmad2/3 might be below the limit of detection, and dephosphorylation within the nucleus may be relatively dominant without a strong exogenous stimulus. For Smad2/3 to enter the nucleus, prior phosphorylation is a requirement [20,45], so it likely that there is increased constitutive Smad2/3 activation in IPF-derived HLMFs. Further experiments will be required to prove this definitively. Similarly, it is likely that K_Ca_3.1 is operating to control αSMA expression via regulation of Smad2/3 signalling, but further experiments involving Smad2/3 downregulation would be required to confirm this.

We used two distinct and selective K_Ca_3.1 blockers at the IC_50_ (20 nM for TRAM-34 and 10 nM for ICA-17043) and at 10× the IC_50_ where >95% of channels will be blocked. These concentrations are physiologically relevant, and furthermore, two structurally similar drugs without channel blocking activity, TRAM-7 and TRAM-85, were without effect here and in previous experiments [22]. Importantly, the concentration of ICA-17043 used here can be achieved in vivo in humans with oral dosing [46], indicating that the targeting of K_Ca_3.1 in IPF is feasible.

## Conclusion

K_Ca_3.1 channel inhibition attenuates many TGFβ1- and bFGF-dependent profibrotic activities in HLMFs [22]. However, as shown here, blocking K_Ca_3.1 channels promotes the de-differentiation of IPF-derived HLMFs towards a quiescent fibroblast phenotype. This suggests that K_Ca_3.1-dependent cell processes may be a common denominator in IPF pathophysiology. K_Ca_3.1 knockout animals are relatively healthy, and the K_Ca_3.1 blocker ICA-17043 (Senicapoc), when delivered orally, was well tolerated for 12 months in a phase III clinical trial of sickle cell disease [46]. Targeting K_Ca_3.1 may therefore provide a novel and effective approach for the treatment of IPF and there is the potential for the rapid translation of K_Ca_3.1-directed therapy to the clinic.

## Abbreviations

IPF: Idiopathic pulmonary fibrosis
NFC: Non fibrotic control
αSMA: α-smooth muscle actin
HLMF: Human lung myofibroblast
TGFβ1: Transforming growth factor Beta 1
TGFβRII: Transforming growth factor beta receptor II
DMEM: Dulbecco’s modified eagle medium
FBS: Fetal bovine serum
IQR: Interquartile range
SEM: Standard error of the mean

## References

[1] Katzenstein AL, Myers JL (1998). Idiopathic pulmonary fibrosis: clinical relevance of pathologic classification. Am J Respir Crit Care Med.

[2] Raghu G, Weycker D, Edelsberg J, Bradford WZ, Oster G (2006). Incidence and prevalence of idiopathic pulmonary fibrosis. Am J Respir Crit Care Med.

[3] Flaherty KR, King TE, Raghu G, Lynch JP, Colby TV, Travis WD, Gross BH, Kazerooni EA, Toews GB, Long Q, Murray S, Lama VN, Gay SE, Martinez FJ (2004). Idiopathic interstitial pneumonia: what is the effect of a multidisciplinary approach to diagnosis?. Am J Respir Crit Care Med.

[4] Raghu G, Collard HR, Egan JJ, Martinez FJ, Behr J, Brown KK, Colby TV, Cordier JF, Flaherty KR, Lasky JA, Lynch DA, Ryu JH, Swigris JJ, Wells AU, Ancochea J, Bouros D, Carvalho C, Costabel U, Ebina M, Hansell DM, Johkoh T, Kim DS, King TE, Kondoh Y, Myers J, Muller NL, Nicholson AG, Richeldi L, Selman M, Dudden RF (2011). An Official ATS/ERS/JRS/ALAT Statement: Idiopathic Pulmonary Fibrosis: Evidence-based Guidelines for Diagnosis and Management. Am J Respir Crit Care Med.

[5] Schwartz DA, Helmers RA, Galvin JR, Van Fossen DS, Frees KL, Dayton CS, Burmeister LF, Hunninghake GW (1994). Determinants of survival in idiopathic pulmonary fibrosis. Am J Respir Crit Care Med.

[6] Gribbin J, Hubbard RB, Le Jeune I, Smith CJ, West J, Tata LJ (2006). Incidence and mortality of idiopathic pulmonary fibrosis and sarcoidosis in the UK. Thorax.

[7] Selman M, King TE, Pardo A, American Thoracic Society, European Respiratory Society, American College of Chest Physicians (2001). Idiopathic pulmonary fibrosis: prevailing and evolving hypotheses about its pathogenesis and implications for therapy. Ann Intern Med.

[8] Tomasek J, Gabbiani G, Hinz B, Chaponnier C, Brown R (2002). Myofibroblasts and mechano-regulation of connective tissue remodelling. Nat Rev Mol Cell Biol.

[9] Sanders YY, Kumbla P, Hagood JS (2007). Enhanced myofibroblastic differentiation and survival in Thy-1(−) lung fibroblasts. Am J Respir Cell Mol Biol.

[10] Hinz B (2007). Formation and function of the myofibroblast during tissue repair. J Invest Dermatol.

[11] Desmouliere A, Geinoz A, Gabbiani F, Gabbiani G (1993). Transforming growth factor-beta 1 induces alpha-smooth muscle actin expression in granulation tissue myofibroblasts and in quiescent and growing cultured fibroblasts. J Cell Biol.

[12] Skalli O, Schurch W, Seemayer T, Lagace R, Montandon D, Pittet B, Gabbiani G (1989). Myofibroblasts from diverse pathologic settings are heterogeneous in their content of actin isoforms and intermediate filament proteins. Lab Invest.

[13] Thannickal VJ, Horowitz JC (2006). Evolving concepts of apoptosis in idiopathic pulmonary fibrosis. Proc Am Thorac Soc.

[14] Kuhn C, McDonald JA (1991). The roles of the myofibroblast in idiopathic pulmonary fibrosis. Ultrastructural and immunohistochemical features of sites of active extracellular matrix synthesis. Am J Pathol.

[15] McAnulty RJ (2007). Fibroblasts and myofibroblasts: their source, function and role in disease. Int J Biochem Cell Biol.

[16] Grinnell F (1994). Fibroblasts, myofibroblasts, and wound contraction. J Cell Biol.

[17] Ellabban NG, Lee KW (1983). Myofibroblasts in Central Giant-Cell Granuloma of the Jaws - an Ultrastructural-Study. Histopathology.

[18] Hu B, Wu Z, Phan SH (2003). Smad3 mediates transforming growth factor-beta-induced alpha-smooth muscle actin expression. Am J Respir Cell Mol Biol.

[19] Gu L, Zhu Y, Yang X, Guo Z, Xu W, Tian X (2007). Effect of TGF-beta/Smad signaling pathway on lung myofibroblast differentiation. Acta Pharmacol Sin.

[20] Nakao A, Imamura T, Souchelnytskyi S, Kawabata M, Ishisaki A, Oeda E, Tamaki K, Hanai J, Heldin CH, Miyazono K, TenDijke P (1997). TGF-beta receptor-mediated signalling through Smad2, Smad3 and Smad4. EMBO J.

[21] Zhou X, Wu W, Hu H, Milosevic J, Konishi K, Kaminski N, Wenzel SE (2011). Genomic Differences Distinguish the Myofibroblast Phenotype of Distal Lung from Airway Fibroblasts. Am J Respir Cell Mol Biol.

[22] Roach K, Duffy S, Coward W, Feghali-Bostwick C, Wulff H, Bradding P (2013). The K^+^ Channel K_Ca_3.1 as a Novel Target for Idiopathic Pulmonary Fibrosis. PLoS ONE.

[23] Huang C, Shen S, Ma Q, Gill A, Pollock CA, Chen X (2014). KCa3.1 mediates activation of fibroblasts in diabetic renal interstitial fibrosis. Nephrol Dial Transplant.

[24] Huang C, Shen S, Ma Q, Chen J, Gill A, Pollock CA, Chen X (2013). Blockade of KCa3.1 ameliorates renal fibrosis through the TGF-beta1/Smad pathway in diabetic mice. Diabetes.

[25] Grgic I, Kiss E, Kaistha BP, Busch C, Kloss M, Sautter J, Muller A, Kaistha A, Schmidt C, Raman G, Wulff H, Strutz F, Grone HJ, Kohler R, Hoyer J (2009). Renal fibrosis is attenuated by targeted disruption of KCa3.1 potassium channels. Proc Natl Acad Sci U S A.

[26] Ramos C, Montaño M, García-Alvarez J, Ruiz V, Uhal BD, Selman M, Pardo A (2001). Fibroblasts from Idiopathic Pulmonary Fibrosis and Normal Lungs Differ in Growth Rate, Apoptosis, and Tissue Inhibitor of Metalloproteinases Expression. Am J Respir Cell Mol Biol.

[27] Keira SM, Ferreira LM, Gragnani A, Duarte IS, Santos, Isabel Anunciação Neves dos (2004). Experimental model for fibroblast culture. Acta Cir Bras.

[28] Pilewski JM, Liu LX, Henry AC, Knauer AV, Feghali-Bostwick CA (2005). Insulin-like growth factor binding proteins 3 and 5 are overexpressed in idiopathic pulmonary fibrosis and contribute to extracellular matrix deposition. Am J Pathol.

[29] Pechkovsky DV, Hackett TL, An SS, Shaheen F, Murray LA, Knight DA (2010). Human Lung Parenchyma but Not Proximal Bronchi Produces Fibroblasts with Enhanced TGF-{beta} Signaling and {alpha}-SMA Expression. Am J Respir Cell Mol Biol.

[30] Zhao J, Shi W, Wang Y, Chen H, Bringas PJ, Datto MB, Frederick JP, Wang X, Warburton D (2002). Smad3 deficiency attenuates bleomycin-induced pulmonary fibrosis in mice. Am J Physiol Lung Cell Mol Physiol.

[31] Wulff H, Miller MJ, Hansel W, Grissmer S, Cahalan MD, Chandy KG (2000). Design of a potent and selective inhibitor of the intermediate-conductance Ca2+−activated K+ channel, IKCa1: a potential immunosuppressant. Proc Natl Acad Sci U S A.

[32] Stocker JW, De Franceschi L, McNaughton-Smith GA, Corrocher R, Beuzard Y, Brugnara C (2003). ICA-17043, a novel Gardos channel blocker, prevents sickled red blood cell dehydration in vitro and in vivo in SAD mice. Blood.

[33] Shumilina E, Lam RS, Wolbing F, Matzner N, Zemtsova IM, Sobiesiak M, Mahmud H, Sausbier U, Biedermann T, Ruth P, Sausbier M, Lang F (2008). Blunted IgE-mediated activation of mast cells in mice lacking the Ca2+−activated K+ channel KCa3.1. J Immunol.

[34] Cruse G, Duffy SM, Brightling CE, Bradding P (2006). Functional KCa3.1 K+ channels are required for human lung mast cell migration. Thorax.

[35] Hu L, Pennington M, Jiang Q, Whartenby KA, Calabresi PA (2007). Characterization of the functional properties of the voltage-gated potassium channel Kv1.3 in human CD4+ T lymphocytes. J Immunol.

[36] Shepherd MC, Duffy SM, Harris T, Cruse G, Schuliga M, Brightling CE, Neylon CB, Bradding P, Stewart AG (2007). K(Ca)3.1 Ca2+−Activated K+ channels regulate human airway smooth muscle proliferation. Am J Respir Cell Mol Biol.

[37] Emblom-Callahan MC, Chhina MK, Shlobin OA, Ahmad S, Reese ES, Iyer EPR, Cox DN, Brenner R, Burton NA, Grant GM, Nathan SD (2010). Genomic phenotype of non-cultured pulmonary fibroblasts in idiopathic pulmonary fibrosis. Genomics.

[38] Bocchino M, Agnese S, Fagone E, Svegliati S, Grieco D, Vancheri C, Gabrielli A, Sanduzzi A, Avvedimento EV (2010). Reactive Oxygen Species Are Required for Maintenance and Differentiation of Primary Lung Fibroblasts in Idiopathic Pulmonary Fibrosis. Plos One.

[39] Coward WR, Watts K, Feghali-Bostwick CA, Knox A, Pang L (2009). Defective histone acetylation is responsible for the diminished expression of cyclooxygenase 2 in idiopathic pulmonary fibrosis. Mol Cell Biol.

[40] Bi D, Toyama K, Lemaitre V, Takai J, Fan F, Jenkins DP, Wulff H, Gutterman DD, Park F, Miura H (2013). The Intermediate Conductance Calcium-activated Potassium Channel KCa3.1 Regulates Vascular Smooth Muscle Cell Proliferation via Controlling Calcium-dependent Signaling. J Biol Chem.

[41] Cruse G, Singh SR, Duffy SM, Doe C, Saunders R, Brightling CE, Bradding P (2011). Functional KCa3.1 K+ channels are required for human fibrocyte migration. J Allergy Clin Immunol.

[42] Di L, Srivastava S, Zhdanova O, Ding Y, Li Z, Wulff H, Lafaille M, Skolnik EY (2010). Inhibition of the K+ channel KCa3.1 ameliorates T cell-mediated colitis. Proc Natl Acad Sci U S A.

[43] Nesti LJ, Caterson EJ, Li W, Chang R, McCann TD, Hoek JB, Tuan RS (2007). TGF-?1 calcium signaling in osteoblasts. J Cell Biochem.

[44] Wicks SJ, Lui S, Abdel-Wahab N, Mason RM, Chantry A (2000). Inactivation of Smad-transforming growth factor beta signaling by Ca2+−calmodulin-dependent protein kinase II. Mol Cell Biol.

[45] Wrighton KH, Lin X, Feng X (2009). Phospho-control of TGF-beta superfamily signaling. Cell Res.

[46] Ataga KI, Smith WR, De Castro LM, Swerdlow P, Saunthararajah Y, Castro O, Vichinsky E, Kutlar A, Orringer EP, Rigdon GC, Stocker JW, ICA-17043-05 Investigators (2008). Efficacy and safety of the Gardos channel blocker, senicapoc (ICA-17043), in patients with sickle cell anemia. Blood.

